This article has been retracted.

# Response of methane production via propionate oxidation to carboxylated multiwalled carbon nanotubes in paddy soil enrichments

**DOI:** 10.7717/peerj.4267

**Published:** 2018-01-12

**Authors:** Jianchao Zhang, Xingxuan Xia, Siliang Li, Wei Ran

**Affiliations:** 1 Institute of Surface-Earth System Science, Tianjin University, Tianjin, China; 2 College of Urban and Environmental Sciences, Peking University, Beijing, China; 3 Jiangsu Provincial Coordinated Research Center for Organic Solid Waste Utilization, Nanjing Agricultural University, Nanjing, China

**Keywords:** Carboxylated, MWCNTs, Syntrophic methanogenesis, Propionate, Anaerobic, Paddy soil enrichment

## Abstract

Carboxylated multiwalled carbon nanotubes (MWCNTs-COOH) have become a growing concern in terms of their fate and toxicity in aqueous environments. Methane (CH_4_) is a major product of organic matter degradation in waterlogged environments. In this study, we determined the effect of MWCNTs-COOH on the production of CH_4_ from propionate oxidation in paddy soil enrichments. The results showed that the methanogenesis from propionate degradation was accelerated in the presence of MWCNTs-COOH. In addition, the rates of CH_4_ production and propionate degradation increased with increasing concentrations of MWCNTs-COOH. Scanning electron microscopy (SEM) observations showed that the cells were intact and maintained their structure in the presence of MWCNTs-COOH. In addition, SEM and fluorescence in situ hybridization (FISH) images revealed that the cells were in direct contact with the MWCNTs and formed cell-MWCNTs aggregates that contained both bacteria and archaea. On the other hand, nontoxic magnetite nanoparticles (Fe_3_O_4_) had similar effects on the CH_4_ production and cell integrity as the MWCNTs-COOH. Compared with no nanomaterial addition, the relative abundances of *Geobacter* and *Methanosarcina* species increased in the presence of MWCNTs-COOH. This study suggests that MWCNTs-COOH exerted positive rather than cytotoxic effects on the syntrophic oxidation of propionate in paddy soil enrichments and affected the bacterial and archaeal community structure at the test concentrations. These findings provide novel insight into the consequences of nanomaterial release into anoxic natural environments.

## Introduction

Carbon nanotubes (CNTs) are hollow cylinders with microscale lengths and nanoscale diameters that are composed of aligned benzene rings (Iijima, 1991). Multi-walled carbon nanotubes (MWCNTs) are widely used due to their unique antimicrobial properties and physicochemical properties including high electrical conductivity, as well as their superior chemical and mechanical stability (De Volder et al., 2013). As a consequence of the rapid increase in the commercial-scale application of MWCNTs, they will accidentally or inevitably enter various environments (Petersen et al., 2011). Release of CNTs could occur at all steps in the life cycle of consumer products. In addition, relevant release scenarios of CNTs are described in detail: injection molding, manufacturing, sports equipment, fuel system components, landfills, windmill blades, electronics, tires, textiles, and incineration (Nowack et al., 2013). Release of CNTs from products can potentially occur by two pathways: (a) where free CNTs are released directly, or (b) where release of particles with CNTs embedded in the matrix (Nowack et al., 2013). For instance, CNTs fate models predict that the CNTs concentrations are between 6.6 ng/L and 18 ng/L in the plant effluent and with a modeled increase in sediment deposition rate of 40 ng/kg to 229 ng/kg per year in United States (Gottschalk et al., 2009).

Biogenic methane (CH_4_) production is carried out by oxygen sensitive methanogenic archaea and hence is restricted to anoxic environments, such as freshwater sediments and rice field soils (Mach et al., 2015). Paddy soil is one of the important natural CH_4_ sources (Conrad, 2009). It is known that interspecies electron exchange is involved in the decomposition of complex organic substances and CH_4_ production in anoxic environments with H_2_ or formate serving as electron carriers (Stams & Plugge, 2009). Recently, direct interspecies electron transfer (DIET) has been proposed as a novel alternative to interspecies electron transfer in methanogenesis (Rotaru et al., 2014a). DIET has been described as cell–cell extracellular electron transfer via electric currents through biological structures (i.e., microbial pili) or abiological conductive solid materials, such as magnetite (Fe_3_O_4_), granular activated carbon and biochar (Liu et al., 2015; Shrestha & Rotaru, 2014). In particular, Fe_3_O_4_, a common iron mineral in soils and sediments, represents a natural material that can accelerate syntrophic CH_4_ production in paddy soil and anaerobic sludge digesters (Kato, Hashimoto & Watanabe, 2012; Li et al., 2015; Liu et al., 2015; Viggi et al., 2014).

Unlike Fe_3_O_4_, granular activated carbon and biochar, MWCNTs have been shown to inhibit the growth and activity of a range of microorganisms in pure culture and exposure to mixed microbial community, including bacteria and protozoa (Kang, Mauter & Elimelech, 2008; Zhao & Liu, 2012). Recent research by Salvador et al. (2017) demonstrated that conductive MWCNTs could accelerate methanogenesis not only by facilitating DIET in the co-cultures from environmental enrichments (Zhang & Lu, 2016) but also in pure cultures of methanogens provided with typical methanogenic substrates. However, it is still unknown how and why methanogenesis gets stimulated by MWCNTs. Furthermore, MWCNTs can potentially be released into the aquatic ecosystem via wastewater discharge and runoff from areas around waste dumps and manufacturing plants, eventually accumulating in the paddy soils or sediments (Farré et al., 2009; Nowack et al., 2013; Petersen et al., 2011). Paddy soil is the most typical and widespread agricultural soil in Asia. In addition, paddy soil represents a hotspot of the CH_4_ emission and production, because the flooded conditions during rice growth (Conrad, 2009). Some studies had shown that MWCNTs had positive effect on the methanogenesis from anaerobic digesters (Ambuchi et al., 2017) and lake sediment (Zhang & Lu, 2016), but the effect of MWCNTs on a methanogenic community from paddy soil has not been previously shown. Propionate is one of the major intermediates in the methanogenic degradation of complex organic matter in paddy soil (Gan et al., 2012). In the present study, to address the possible influence of carboxylate-functionalized MWCNTs (MWCNTs-COOH) on syntrophic methanogenesis from propionate oxidation, methanogenic communities were enriched from paddy soil in the presence and absence of MWCNTs-COOH. Fluorescence *in situ* hybridization (FISH) and scanning electron microscopy (SEM) were used to visualize the interactions between microbial cells and MWCNTs-COOH. The effect of MWCNTs-COOH on the microbial consortia was also investigated. The results of this study will provide useful information to understand the response of methanogenic communities to MWCNTs-COOH in paddy soil.

## Materials and Methods

### Nanomaterial preparation and characterization

Commercially available carboxylic (-COOH) functionalized MWCNTs were purchased from DK Nano Technology Co. (Beijing, China). According to the manufacturer, the purity was more than 99% by mass, the average diameter and length of MWCNTs-COOH were approximately 10–20 nm and 10–30 µm, and the COOH content was approximately 2% (w/w). A ten percent (w/v) MWCNTs-COOH stock water suspension was used for the experiments. Nano-sized Fe_3_O_4_ particles (50–100 nm) were purchased from Sigma-Aldrich (637106; St. Louis, MO, USA).

### Inoculum source and anaerobic media

Flooded paddy soil was collected from Tianjin, northern China (43°44′N 126°30′E). The soil had the following characteristics: total organic carbon content of 1.90%, total nitrogen content of 0.12% and pH (H_2_O) 7.85. The soil is classified as a clay texture. The soil samples were collected in July 2016 at a depth of 0–20 cm. Twelve soil cores (approximately 5 cm in diameter) were taken from the flooded paddy field and mixed to form one composite sample. Soil samples were placed in sealed bottles that were filled and transported to the lab as soon as possible. The soil samples were stored at 4 °C until use.

HEPES-buffered (30 mM, pH 7) anaerobic basal medium was used for enrichment and subsequent transfers. The basal medium preparation followed a previously described protocol (Lü & Lu, 2012). Sodium propionate was added as a substrate at a final concentration of 10 mM through injection via an aseptic syringe into the bottled culture medium. A concentration of up to 10 mM propionate can be locally found during the anaerobic decomposition of organic matter (Gan et al., 2012).

### Enrichment procedures

For the initial enrichment (first enrichments), approximately 5 g of fresh soil (2.13 g dry soil) was transferred in triplicate into sterile 120 ml serum bottles filled with 40 ml of medium and closed with butyl rubber stoppers. Four treatments were conducted in the enrichments, including a no nanomaterial supplementation control treatment (CK-1), MWCNTs-COOH supplementation treatment 1 (MWCNTs-COOH-1, final concentration of 1 g/L), MWCNTs-COOH treatment 2 (MWCNTs-COOH-2, final concentration of 0.1 g/L) and nanoFe_3_O_4_ supplementation treatment (the final concentration of 10 mM as Fe atom). The addition of electrically conductive Fe_3_O_4_ nanoparticles (natural occurring mineral in environments) was used as positive control for evaluating the effects from MWCNTs-COOH.

When the CH_4_ production from the MWCNTs-COOH treatment 1 approached a plateau, a portion of the culture from the MWCNTs-COOH treatment 1 was transferred to a bottle containing 40 ml of fresh medium (next enrichment culture) (Figure S1). For all the transfers in this study, the inoculum size was 4% (v/v). Four treatments with inocula from MWCNTs-COOH-1 were performed for the subsequent enrichments. The first and fourth transfers are only shown in the present study because the first to fourth enrichments behaved similarly. In addition, another batch of enrichments (CK-2) was conducted simultaneously with inocula from the no nanomaterial supplementation treatment (Figure S1). The schematic diagram of the experimental design is shown in Fig. 1. All the enrichments were incubated statically in the dark at 30 °C under an atmosphere of N_2_/CO_2_ [80:20 (V/V)].

**Figure 1:** Effects of MWCNTs-COOH and Fe_3_O_4_ supplementation on the production of CH_4_ (A, B) and the degradation of propionate (C, D) for the first and fourth enrichments. Error bars represent the standard deviation of three replicates. MWCNTs-1: MWCNTs-COOH supplementation treatment 1 with a final concentration of 1 g/L; MWCNTs-2: MWCNTs-COOH supplementation treatment 2 with a final concentration of 0.1 g/L.

### Chemical analyses

The CH_4_ concentration was analysed using a gas chromatograph (7890; Agilent Technologies, Santa Clara, CA, USA) equipped with flame ionization detector (FID) (Peng et al., 2008). Gas samples (100 µl) were collected from the headspace using a Pressure-Lok precision analytical syringe (Bation Rouge, LA USA) every two to five days. Liquid samples (0.5 ml) were collected every four to nine days with a sterile syringe, centrifuged, and filtered through 0.22 µm filters (Millipore, Burlington, MA, USA). The concentrations of propionate were analysed by high-pressure liquid chromatography (HPLC) with a Zorbax SB-AQ C18 column (Agilent Technologies, Santa Clara, CA, USA) (Krumböck & Conrad, 1991).

### Microscopy analysis

The cultures in the fourth enrichments were subjected to microscopy when the cell communities were enriched. The cells in the CK-1, Fe_3_O_4_ and MWCNTs-1 treatments were collected using a sterile syringe, fixed with 2.5% (wt/vol) glutaraldehyde in phosphate-buffered saline, and sequentially dehydrated with serial ethanol dilutions (20, 40, 60, 80, 95 and 100% (v/v) with every 10 min per step). The dried samples were coated with platinum and imaged using scanning electron microscopy (FEI NanoSEM 430).

In addition, fluorescence *in situ* hybridization (FISH) analysis was performed on 4% paraformaldehyde-fixed samples according to a procedure described previously (Moter & Göbel, 2000). Oligonucleotide probes specific for bacteria (Cy3-labeled EUB338mix probes) and archaea (FITC-labeled ARC915 probe) were used in this study. The details of the probes used are available in probeBase (http://probebase.csb.univie.ac.at/) (Greuter et al., 2016). The labelled samples were visualized using epifluorescence microscopy (Axio Imager D2; ZEISS, Oberkochen, Germany).

### Molecular analysis of the microbial community

The cells in the MWCNTs-COOH-1 and CK-2 treatments were harvested from triplicate cultures at the fourth enrichments. In addition, the cells from different treatments were collected in the mid-log phase (CH_4_ concentration about 12 mM) by syringe. Total DNA was extracted using the FastDNA SPIN Kit (MP Biomedicals, Santa Ana, CA, USA) according to the manufacturer’s protocol. Prior to DNA extraction, sonication was performed to separate the microbial cells from the MWCNTs. The DNA was extracted from each replicate and stored at −20 °C.

We used high throughput Miseq sequencing for the analysis of the microbial community in the enriched cultures. The V3–V4 universal primers 314F/805R were used to determine the bacterial communities. In addition, the 349F/806R primers were used to amplify the archaeal 16S rRNA genes. Sequencing was performed using the Illumina Miseq 2 × 300 bp platform (San Diego, CA, USA) by Sangon Biotech Company (Shanghai, China).

We used the Quantitative Insights Into Microbial Ecology (QIIME) (Caporaso et al., 2010) and UPARSE pipeline (Edgar, 2013) to treat the raw sequencing data. Barcodes and standard primer sets were excluded. The UPARSE pipeline was used to select the operational taxonomic units (OTUs), and the sequences were assigned to OTUs with 97% similarity. Then, a representative OTU sequence was assigned to a taxonomic identity using RDP classifier (http://rdp.cme.msu.edu) (Wang et al., 2007) with a default confidence threshold of 0.8–1.0. Raw sequencing reads have been deposited into the NCBI SRA with the accession number SRP108450.

## Results

### Effects of MWCNTs-COOH on CH_4_ production

The effect of MWCNTs-COOH on CH_4_ production by methanogenic enrichment cultures was assessed (Fig. 1). Two enrichments (first and fourth) were revealed in the present study because the first to fourth enrichments behaved similarly. In the incubations, the results showed that the addition of Fe_3_O_4_ and MWCNTs-COOH increased the rate of methane production from propionate oxidation. In addition, CH_4_ production at a MWCNTs-COOH concentration of 1 g/L was faster than that at 0.1 g/L (Figs. 2A, 2B). In the first enrichments (Fig. 1A), the time preceding the completion of CH_4_ production was much shorter in the assays with Fe_3_O_4_ and with high concentration of MWCNTs-COOH (approximately 31 days) than in the assays without nanomaterials (approximately 46 days) or with low concentration of MWCNTs-COOH (approximately 42 days). The production of CH_4_ in the fourth enrichment cultures was faster than the first enrichments for all the treatments, but the stimulating effect of MWCNTs and Fe_3_O_4_ remained evident.

**Figure 2:** Spatial distribution of archaeal (Arc915-FITC, green) and bacterial (EUB338mix-Cy3, red) cells identified by FISH in enrichments with CK-1 (A), Fe_3_O_4_ (B) and MWCNTs-1 (C) treatments. Cell aggregates were formed irrespective of the treatment. Blurry black plots with red or dark backgrounds within the cell aggregates (indicated by white arrows) could be found in the presence of Fe_3_O_4_ and MWCNTs-COOH.

Similarly, propionate conversion to CH_4_ was also enhanced by the presence of Fe_3_O_4_ and MWCNTs (Figs. 1C, 1D). In the first enrichment cultures, propionate degradation in the assays with Fe_3_O_4_ and high concentration of MWCNTs-COOH started after a shorter lag phase and proceeded to completion more rapidly compared to the assays without nanomaterials or with low concentration of MWCNTs-COOH (36 days vs 42 or 46 days). Subsequent enrichments showed similar trends to those in the first enrichments.

In the incubations, approximately 17.8 mM CH_4_ was produced from 10.1 mM propionate (Fig. 1). This result suggests that the syntrophic interaction in the enrichments followed the stoichiometry of the complete conversion of propionate to CH_4_ (4CH_3_CH_2_COO^−^ + 4H^+^ + 2H_2_O → 7CH_4_ + 5CO_2_).

### FISH assays

The FISH images exhibited strong fluorescence bacterial (in red) and archaeal (in green) signatures in the enrichments, indicating that the cells in the MWCNTs-COOH treatment were active and intact as in the CK-1 and Fe_3_O_4_ treatments (Fig. 2). Classical *Sarcina*-like shapes were dominant with filamentous cells accounting for a small fraction in the archaeal cells (Fig. 2). In addition, we found that numerous aggregates were formed irrespective of the treatment. FISH observations revealed that the bacteria were in close contact with the archaeal cells in the aggregates.

### SEM observations

Abundant aggregates were also observed by SEM (Fig. 3). In addition to short-rod and long slender-rod cells, the *Sarcina*-like cells were dominant. The bacterial and archaeal cells in the control were in close contact forming dense microbial aggregates (Fig. 3A). In the MWCNTs-COOH-1 treatment, however, most of the cells were in association with MWCNTs-COOH and formed cells-nanomaterial mixtures (Figs. 3C, 3D). Though microbial cells appeared more separated in MWCNTs-COOH compared with those with close physical proximity in the control, most of the microbial cells were interconnected by the MWCNTs-COOH. SEM observations of the enrichments where MWCNTs-COOH was replaced with nanoFe_3_O_4_, which had similar architecture to the microbe-nanomaterial hybrid aggregates (Fig. 3B).

**Figure 3:** Interactions between microbial cells and nanomaterials (MWCNTs-COOH and Fe_3_O_4_) in the enrichment treatments by scanning electron micrographs (SEM). CK-1: (A); Fe_3_O_4_: (B); MWCNTs-1: (C, D). White arrows (B, C and D) indicate Fe_3_O_4_ nanoparticles or MWCNTs-COOH.

In addition, the SEM images showed that the cells in the MWCNTs-COOH treatment were intact and maintained their structure, similar to the cells in the control and nanoFe_3_O_4_ treatments. These results indicated that no obvious cellular damage occurred when the cells were in contact with high concentration (1 g/L) of MWCNTs-COOH.

### Microbial community compositions

Analysis of the microbial communities was carried out for the fourth enrichments with the MWCNTs-COOH-1 and CK-2 treatments. In the MWCNTs-COOH-1 enrichment, the 16S rRNA gene sequencing revealed that the bacterial populations were dominated by *Smithella* (24%) and *Syntrophomonas* (19%), followed by *Geobacter* (14%), *Syntrophobacter* (9%), *Clostridium* (6%), *Pelotomaculum* (7%), *Desulfobulbus* (3.7%) and *Sulfurospirillum* (3.1%) (Fig. 4A). The archaeal community (Fig. 4B) in the MWCNTs-COOH-1 enrichment consisted mainly of *Methanosarcina* (44%) and *Methanoregula* (16%), with a minor proportion of *Methanosaeta* (12%), *Methanocella* (4%), *Methanomicrobium* (5%) and *Methanobacterium* (4%). By comparison, the predominant bacterial components in the CK-2 enrichment (Fig. 4A) consisted of *Syntrophobacter* (23%), *Pelotomaculum* (18%) *Smithella* (19%) and *Syntrophomonas* (11%) with a minor proportion of *Clostridium* (3%) and *Geobacter* (4%). In addition, the archaeal community in the CK-2 enrichment consisted of *Methanosarcina* (27%), *Methanoregula* (11%) *Methanosaeta* (8%), *Methanocella* (18%), *Methanomicrobium* (9%), *Methanobacterium* (15%).

**Figure 4:** The phylogenetic classification and relative abundance of the bacteria (A) and archaea (B) at the genus level in the enrichments of the MWCNTs-1 and CK-2 treatments. “Other” indicates the genus of the bacteria (A) or archaea (B) with a low relative abundance (less than 2%). The error bars represent standard deviations from the triplicate samples of each treatment.

## Discussion

### MWCNTs-COOH and the cell damages

MWCNTs have been reported to cause different inhibitory effects on microorganisms (Kang, Mauter & Elimelech, 2008; Yadav, Mungray & Mungray, 2016). Previous SEM studies showed that CNT-treated cells lost their cellular integrity (flattened or misshapen) (Kang, Mauter & Elimelech, 2008). The antimicrobial mechanism probably involves oxidative stress and cell membrane damage (Du et al., 2013). Additionally, the results from Kang et al. (2007) suggested that physical interaction of CNTs with bacterial cells, rather than oxidative stress, is the primary killing mechanism. Otherwise, the antimicrobial activity of CNTs was regulated by their concentration (Das et al., 2014). In the current study, relatively high concentration of MWCNTs-COOH (1 g/L) was applied compared to previous studies on the inhibitory effects (Nouara et al., 2013; Wang et al., 2014). If the inhibitory mechanisms worked, more severe effects would be anticipated in the present experiment. However, we did not observe adverse effects in this study. Instead, the effects of MWCNTs-COOH on CH_4_ production from propionate degradation were positive in our enrichments, similar to the effects of Fe_3_O_4_. Furthermore, the acceleration of CH_4_ production was higher with the highest MWCNTs concentration tested (Fig. 1). FISH observations suggested that the bacterial and archaeal cells were aggregated irrespective of the treatment (Fig. 2). SEM images further verified the formation of cell-MWCNTs aggregates in the MWCNTs treatment and showed that the cells were in direct contact with the MWCNTs (Fig. 3). According to our SEM observations, penetration into the cell membranes or adverse effects on the cellular integrity did not occur.

The lack of inhibitory effect in the present experiment was probably due to the anaerobic conditions. Oxidative stress by MWCNTs resulted from the production of reactive oxygen species (ROS) due to the small size and high reactivity of MWCNTs (Du et al., 2013). It was also shown that the MWCNTs-COOH could generate notable amounts of ROS during UVA irradiation at an intensity similar to that in the sunlight (Qu, Alvarez & Li, 2013). However, the enrichment cultivation in the present experiment was carried out in the dark and under anaerobic conditions. Thus, oxidative stress should not be a significant factor in this study. In addition, the cytotoxicity of CNTs is often attributed to the physicochemical properties of CNTs. The carboxylate functionalization of MWCNTs is thought to make the nanomaterials more biocompatible than the pristine MWCNTs due to their improved hydrophilicity and dispersion in the biological media (Vardharajula et al., 2012). The CNTs used in this study are carboxylated MWCNTs.

### MWCNTs-COOH and microbial community in the syntrophic consortia

Instead of inhibition, the addition of MWCNTs-COOH substantially facilitated the syntrophic production of CH_4_ from propionate oxidation. Stimulation of CH_4_ production in the presence of Fe_3_O_4_ has been reported previously (Kato, Hashimoto & Watanabe, 2012; Li et al., 2015; Liu et al., 2015; Rotaru et al., 2014a; Viggi et al., 2014; Zhang & Lu, 2016). All the existing reports suggested the Fe_3_O_4_ acts as a conductor that facilitates or accelerates the transfer of electrons between *Geobacter* and acetotrophic methanogens (*Methanosarcina* and *Methanosaeta*). *Geobacter* species are widespread in anoxic soils and typically carry out a dissimilatory reduction on extracellular electron acceptors, such as Fe(III), coupled with the oxidation of acetate and other electron donors (Mahadevan, Palsson & Lovley, 2011; Richter, Schicklberger & Gescher, 2012). Previous studies have demonstrated that *Geobacter* could participate in the syntrophic oxidation of propionate in the paddy soil under methanogenic conditions by stable-isotope probing (Gan et al., 2012; Lueders, Pommerenke & Friedrich, 2004). The microbial mechanisms of DIET between *Geobacter* and methanogens were extensively studied (Holmes et al., 2017; Liu et al., 2012; Morita et al., 2011; Rotaru et al., 2014a; Rotaru et al., 2014b). Electrical connections that support the DIET capacity of *Geobacter* include electrically conductive pili (e-pili) and cytochromes. The presence of *Geobacter* species is often equated with the occurrence and capacity for DIET (Holmes et al., 2017). Compared with CK-2, the relative abundance of *Geobacter* was increased in the presence of MWCNTs-COOH and accounted for 14% of the bacterial community (Fig. 4). In addition, *Methanosarcina* was large enriched in the presence of MWCNTs-COOH. Previous studies also showed that the abundance of *Geobacter* species as well as the conductive materials, simultaneously enhance the growth of *Geobacter* and the CH_4_ production in the methanogenic soils (Kato, Hashimoto & Watanabe, 2012; Li et al., 2015; Rotaru et al., 2015). Owing to the high electrical conductivity of MWCNTs-COOH, it seems that MWCNTs-COOH have a similar function with Fe_3_O_4_ to facilitate DIET in syntrophic methanogenesis from propionate. However, in this study, we did not have sufficient evidence to support the occurrence of DIET in the syntrophic consortia from propionate oxidation. In particular, the study from Salvador et al. (2017) suggested that CNTs significantly accelerated the CH_4_ production directly by pure methanogens and that the direct effect was independent of possible mechanisms, such as DIET. Convincing mechanisms for the simulation of CH_4_ production from propionate oxidation are still unknown. Elucidation of the mechanisms that enhance CH_4_ production will require much more extensive investigation with novel approaches in future work.

Recent studies showed that CNTs could also stimulate CH_4_ production in lake sediments with butyrate oxidation, anaerobic rectors with beet sugar digestion and pure cultures of methanogens (Ambuchi et al., 2017; Salvador et al., 2017; Zhang & Lu, 2016). However, the effect of MWCNTs-COOH on the syntrophic consortia from propionate oxidation in paddy soil enrichment was never reported. Our study verified that the MWCNTs-COOH could change the relative abundance of the dominant bacterial and archaeal genera in paddy soil enrichment (Fig. 4). *Smithella* utilize propionate in a nonrandomizing pathway in which propionate is first dismulated to acetate and butyrate before being degraded via β-oxidation, while *Syntrophomonas* are known butyrate degraders (Dolfing, 2013; Gan et al., 2012; Lueders, Pommerenke & Friedrich, 2004). There were increases in the relative abundances of the bacterial genera such as *Geobacter*, *Smithella*, *Syntrophomonas* and the archaeal genera such as *Methanosarcina* in the MWCNTs-COOH treatment*.* However, there were no significant differences in the bacterial and archaeal community compositions during the enrichment. Recent studies also showed that microbe community structure significantly shifted after CNTs addition (Ambuchi et al., 2017; Shrestha et al., 2013; Zhang & Lu, 2016). For example, the bacterial genera such as *Rhodococcus*, *Cellulomonas* and *Nocardioides* were increased after the addition of 1 g/kg MWCNTs in sandy loam soil (Shrestha et al., 2013). In addition, the fungal genera *Pseudeurotium* and *Penicillium* (important in the soil carbon and phosphorus biogeochemical cycling) were decreased after the addition of 0.5 g/kg CNTs into a grass soil (Rodrigues, Jaisi & Elimelech, 2013).

By 2011, the worldwide CNTs production had jumped to about 4.6 kilotons per year (De Volder et al., 2013). As they are adopted for increasing use in consumer products, there is a potential for CNTs to enter the environment through both accidental discharge and intentional application. Potential CNTs release mechanisms during the CNTs/polymer lifecycle include biodegradation, washing, diffusion, matrix degradation and incineration (Petersen et al., 2011). While many previous studies have been focused on the toxicity of these materials to microorganisms and human health, our study prompts further investigation to evaluate the various consequences of nanomaterial release into anoxic natural environments.

## Conclusions

The supplementation of MWCNTs-COOH displayed a substantial stimulatory effect on anaerobic syntrophic CH_4_ production in paddy soil enrichment. MWCNTs-COOH exerted positive, rather than cytotoxic, effects on the microbes involved in syntrophic methanogenesis from propionate degradation and affected the bacterial and archaeal community structure in the test concentrations.

##  Supplemental Information

10.7717/peerj.4267/supp-1 Figure S1 Schematic diagram of the experimental design with different treatments Two batches of enrichments were performed in this study with different inocula: the cells from all the MWCNTs-COOH treatment or no nanomaterial supplementation control, respectively. MWCNTs-1: MWCNTs-COOH supplementation treatment 1 with a final concentration of 1 g/L; MWCNTs-2: MWCNTs-COOH supplementation treatment 2 with a final concentration of 0.1 g/L. The cultures in the fourth enrichment were subjected to microscopy and molecular phylogenetic analyses.

## Additional Information and Declarations

### Data Availability

The following information was supplied regarding data availability: NCBI: SRP108450.
